# Morphological Reconstruction-Based Image-Guided Fuzzy Clustering with a Novel Impact Factor

**DOI:** 10.1155/2021/6747371

**Published:** 2021-09-13

**Authors:** Qingxue Qin, Guangmei Xu, Jin Zhou, Rongrong Wang, Hui Jiang, Lin Wang, Shiyuan Han, Tao Du, Ke Ji, Ya-ou Zhao, Kun Zhang

**Affiliations:** ^1^Shandong Provincial Key Laboratory of Network Based Intelligent Computing, University of Jinan, Jinan 250022, China; ^2^Department of Internet Business, Shandong Technician Institute, Jinan 250200, China; ^3^Development and Test Center, Chinabond Fintech Information Technology Co. Ltd., Beijing 100032, China

## Abstract

The guided filter is a novel explicit image filtering method, which implements a smoothing filter on “flat patch” regions and ensures edge preserving on “high variance” regions. Recently, the guided filter has been successfully incorporated into the process of fuzzy c-means (FCM) to boost the clustering results of noisy images. However, the adaptability of the existing guided filter-based FCM methods to different images is deteriorated, as the factor *ε* of the guided filter is fixed to a scalar. To solve this issue, this paper proposes a new guided filter-based FCM method (IFCM_GF), in which the guidance image of the guided filter is adjusted by a newly defined influence factor *ρ*. By dynamically changing the impact factor *ρ*, the IFCM_GF acquires excellent segmentation results on various noisy images. Furthermore, to promote the segmentation accuracy of images with heavy noise and simplify the selection of the influence factor *ρ*, we further propose a morphological reconstruction-based improved FCM clustering algorithm with guided filter (MRIFCM_GF). In this approach, the original noisy image is reconstructed by the morphological reconstruction (MR) before clustering, and the IFCM_GF is performed on the reconstructed image by utilizing the adjusted guidance image. Due to the efficiency of the MR to remove noise, the MRIFCM_GF achieves better segmentation results than the IFCM_GF on images with heavy noise and the selection of the influence factor for the MRIFCM_GF is simple. Experiments demonstrate the effectiveness of the presented methods.

## 1. Introduction

Image segmentation is considered an indispensable component in image processing, comprehension, and computer vision [1–3]. In the last few decades, prototype-based clustering has been broadly applied in image segmentation [4–6]. Owing to the inherent vagueness of the image, fuzzy clustering, such as FCM, can achieve better performance in image segmentation tasks than hard clustering [7, 8].

However, because the FCM-based image segmentation methods only reflect the intensity of the pixel itself, they are ineffective when images are corrupted by noise [9, 10]. To solve this issue, a novel FCM approach with spatial constraints (FCM_S) is developed in [11], which partitions a pixel into a cluster according to both the intensity value of itself and the ones of its neighbor pixels. However, FCM_S needs to spend countless time to compute the spatial neighbor term. To alleviate the computation time in the FCM_S, two improved versions (FCM_S1 and FCM_S2) are explored by utilizing average filter and median filter to attain the spatial information beforehand [12]. The two aforementioned clustering algorithms with spatial constraints are robust to noise, but they get poor segmentation results on the image edges [11–13]. This is because the computation of spatial information smooths the whole image and leads to the damage of boundary information.

Then, the guided filter is considered to address this issue, which not only implements a smoothing filter on “flat patch” regions to relieve the impacts of noise but also ensures edge preserving on “high variance” regions [14, 15]. The image-guided FCM (IGFCM) method is exploited by adding a guided filter to the optimization of FCM [16], but the complexity of the IGFCM model leads to vast calculation time. To tackle this problem, a new method called FCM + GF is further developed in [17], in which the FCM is employed to segment the raw noise image and the guided filter is implemented on the membership metrics by adopting the raw noise image as the guidance. This method achieves good segmentation results with low computational complexity. Nevertheless, in FCM + GF, the factor *ε* regarding guided filter is fixed to a scalar, which deteriorates the capability of FCM + GF to divide images in the case of various noise rates. Actually, the value of *ε* is considered to differ with the increase of the noise level.

In this paper, a guided filter-based FCM algorithm with an impact factor named IFCM_GF is presented, in which a novel positive impact factor *ρ* is defined to adapt the guidance image. This adjustment on the guidance image is proved to be equivalent to the change of parameter *ε*. Given different *ρ*, the IFCM_GF obtains better performance on various noisy rates images than FCM + GF with the fixed *ε*.

However, there are still two shortcomings of the IFCM_GF. The first one is that it is uneasy to choose an appropriate value *ρ* empirically because the good value of *ρ* varies according to different noise rates. The second one is that the IFCM_GF is not robust to noise type and obtains poor segmentation results on the images with heavy noise. This is because both the image to be partitioned and the image to provide guidance information are the original noisy image. To overcome the above two shortcomings simultaneously, we introduce morphological reconstruction (MR) [18] to the IFCM_GF and propose a morphological reconstruction-based improved FCM clustering algorithm with guided filter, named MRIFCM_GF. In the approach, the FCM is conducted on the reconstructed image obtained by MR, and the guided filter is implemented on the membership metrics with the guidance of the raw noise image adjusted by the impact factor *ρ*. The MR adopts a marker image to recast raw noise image so as to acquire a better image [19]. On the one hand, there is a little difference between the reconstructed images of the original images with different noise rates, so it is easier to set a good *ρ* for MRIFCM_GF. On the other hand, since MR can remove noise without knowing the type of noise and preserve the edge information of image, MRIFCM_GF can achieve better performance on images with heavy noise than IFCM_GF. What is more, as the reconstructed image is calculated beforehand, the employment of the MR brings little extra calculation time. The main contributions of this paper are briefly summarized as follows.

Firstly, the IFCM_GF method with a newly defined factor *ρ* is proposed to enhance the adaptability for different noisy images.

Secondly, the MRIFCM_GR method is further developed by incorporating MR technique into IFCM_GF for better segmentation performance on images with heavy noise and easier selection of proper values of factor *ρ*.

The rest part of this paper is organized as follows. Some related works are reviewed in Section 2. The presented algorithms and the proof are detailed in Section 3. The experiments are elaborated in Section 4. Finally, Section 5 summarizes the conclusion.

## 2. Related Works

### 2.1. Fuzzy C-Means

FCM is a prototype-based clustering approach which is extensively applied in image segmentation. Let {*x*_*n*_, *n*=1,2, ..., *N*} stand for *N* pixels in an image, *C* indicates the number of clusters, and FCM partitions the *N* pixels into *C* clusters by solving the following minimization problem:

(1) $$\begin{array}{c} J\left(U,V\right)=\sum_{c=1}^{C}\sum_{n=1}^{N}u_{cn}^{m}{\left\|x_{n}-v_{c}\right\|}^{2},\\ \text{subject to}\;\sum_{c=1}^{C}u_{cn}=1,\;0<u_{cn}<1, \end{array}$$

where *U*=[*u*_*cn*_] is the membership degree matrix and *u*_*cn*_ means the membership of pixel *x*_*n*_ in cluster *c*. *V*=[*v*_*c*_] denotes the cluster prototype matrix, and *v*_*c*_ denotes the center vector of cluster *c*. The parameter *m*(*m* > 1) indicates the fuzzification index, and the norm ‖·‖ represents the Euclidean norm.

Minimizing *J*(*U*, *V*) is a nonlinear optimization problem with a constraint. The Picard iteration is used to solve it. First, *V* is fixed to find *U* minimizing *J*(*U*). Then, *U* is fixed to find V minimizing *J*(*V*).

When *V* is fixed, the Lagrange multiplier technique is applied to convert the min *J*(*U*, *V*) into an unconstrained optimization problem regarding *U* asfollows:

(2) $$\begin{array}{c} \tilde{J}\left(U,\Lambda \right)=\sum_{c=1}^{C}\sum_{n=1}^{N}u_{cn}^{m}{\left\|x_{n}-v_{c}\right\|}^{2}-\sum_{n=1}^{N}\lambda_{n}\left(\sum_{c=1}^{C}u_{cn}-1\right), \end{array}$$

where Λ=[*λ*_*n*_] is a Lagrange multipliers matrix corresponding to the constraint ∑_*c*=1_^*C*^*u*_*cn*_=1. Set the partial derivatives of *J*(*U*, Λ) regarding *u*_*cn*_ and *λ*_*n*_ to zero as follows:

(3) $$\begin{array}{c} \frac{\partial J\left(U,\Lambda \right)}{\partial u_{cn}}=mu_{cn}^{m-1}{\left\|x_{n}-v_{c}\right\|}^{2}-\lambda_{n}=0, \end{array}$$

(4) $$\begin{array}{c} \frac{\partial J\left(U,\Lambda \right)}{\partial \lambda_{n}}=-\left(\sum_{c=1}^{C}u_{cn}-1\right)=0. \end{array}$$

From, (3) and (4), (5) is obtained.

(5) $$\begin{array}{c} u_{cn}=\frac{1}{\sum_{j=1}^{C}{\left(\left\|x_{n}-v_{c}\right\|/\left\|x_{n}-v_{j}\right\|\right)}^{\left(2/\left(m-1\right)\right)}}, \end{array}$$

for 1 ≤ *c* ≤ *C*,  1 ≤ *n* ≤ *N*.

When *U* is fixed, set the gradient of *J*(*V*) with respect to *v*_*c*_ to zero to make *J*(*V*) locally minimized as follows:

(6) $$\begin{array}{c} \frac{\partial J\left(V\right)}{\partial v_{c}}=-2\sum_{n=1}^{N}u_{cn}^{m}\left(x_{n}-v_{c}\right)=0. \end{array}$$

From (6), (7) is obtained.

(7) $$\begin{array}{c} v_{c}=\frac{\sum_{n-1}^{N}u_{cn}^{m}x_{n}}{\sum_{n-1}^{N}u_{cn}^{m}}, \end{array}$$

for 1 ≤ *c* ≤ *C*, 1 ≤ *n* ≤ *N*.

Equations (5) and (7) are repeatedly implemented until the difference between the optimization problem regarding two successive iterations is small enough.

### 2.2. Guided Filter

Guided filter is widely utilized in linear filtering area. Considering an input image *p* and the guidance image *I*, the output image *q* is obtained as follows:

(8) $$\begin{array}{c} q_{i}=a_{k}I_{i}+b_{k},\;\forall_{i}\in \omega_{k}, \end{array}$$

where *i* and *k* are pixel indexes and *ω*_*k*_ denotes a window centralized at the pixel *k*. *a*_*k*_ and *b*_*k*_ indicate some linear scalars with respect to the pixel of *ω*_*k*_. This local linear model is able to preserve the edge information due to ∇*q*=*a*∇*I*. And the capability of this model is proved in image processing.

To get the linear coefficients, the minimization of the difference between the input image *p* and the output image *q* is adopted to establish the cost equation as follows:

(9) $$\begin{array}{c} E\left(a_{k},b_{k}\right)=\sum_{i\in \omega_{k}}\left({\left(a_{k}I_{i}+b_{k}-p_{i}\right)}^{2}+\varepsilon a_{k}^{2}\right), \end{array}$$

where *ε* indicates a regularized indicator to prevent *a*_*k*_ from being too big.

Let the gradients of *E*(*a*_*k*_, *b*_*k*_) regarding *a*_*k*_ and *b*_*k*_ be equal to zero as follows:

(10) $$\begin{array}{c} \frac{\partial E}{\partial a_{k}}=\sum_{i\in \omega_{k}}\left(2\left(a_{k}I_{i}+b_{k}-p_{i}\right)I_{i}+2\varepsilon a_{k}\right)=0, \end{array}$$

(11) $$\begin{array}{c} \frac{\partial E}{\partial b_{k}}=\sum_{i\in \omega_{k}}2\left(a_{k}I_{i}+b_{k}-p_{i}\right)=0. \end{array}$$

From (10) and (11), *a*_*k*_ and *b*_*k*_ are obtained as follows:

(12) $$\begin{array}{c} a_{k}=\frac{\left(1/\left|\omega \right|\right)\sum_{i\in \omega_{k}}I_{i}p_{i}-\mu_{k}\bar{p_{k}}}{\sigma_{k}^{2}+\varepsilon }, \end{array}$$

(13) $$\begin{array}{c} b_{k}=\bar{p_{k}}-a_{k}\mu_{k}, \end{array}$$

where |*ω*| denotes the number of pixels, *μ*_*k*_ and *σ*_*k*_ indicate the mean and variance of *I*, and $\bar{p_{k}}$ represents the mean of *p* in window *ω*_*k*_.

*a*_*k*_ and *b*_*k*_ are associated with the window *ω*_*k*_, so *q*_*i*_ may be different when calculated in different *ω*_*k*_. The final output *q*_*i*_ is the average of all the possible values and is computed as follows:

(14) $$\begin{array}{c} q_{i}=\frac{1}{\left|\omega \right|}\sum_{k:i\in \omega_{k}}a_{k}I_{i}+b_{k}=\bar{a_{i}}I_{i}+\bar{b_{i}}, \end{array}$$

where $\bar{a_{i}}=\left(1/\left|\omega \right|\right)\sum_{k\in \omega_{i}}a_{k}$ and $\bar{b_{i}}=\left(1/\left|\omega \right|\right)\sum_{k\in \omega_{i}}b_{k}$.

### 2.3. Morphological Reconstruction

As an effective method for image denoising and edge preservation simultaneously, morphological reconstruction includes two basic operations, that is, morphological dilation and erosion reconstructions.

Morphological dilation is defined as

(15) $$\begin{array}{c} R_{f}^{\delta }\left(g\right)=\delta_{f}^{n}\left(g\right), \end{array}$$

where *f* denotes the mask image, *g* indicates the marker image and *g* ≤ *f*, *δ* denotes the dilation operator, and *δ*_*f*_^1^(*g*)=*δ*(*g*)∧*f*,  *δ*_*f*_^*n*^(*g*)=*δ*_*f*_^1^(*δ*_*f*_^*n*−1^(*g*))∧*f*, ∧ represents the pointwise minimum.

Morphological erosion is defined as

(16) $$\begin{array}{c} R_{f}^{\varepsilon }\left(g\right)=\varepsilon_{f}^{n}\left(g\right), \end{array}$$

where *g* ≥ *f*, *ε* denotes erosion operator, and *ε*_*f*_^1^(*g*)=*ε*(*g*)∨*f*, *ε*_*f*_^*n*^(*g*)=*ε*_*f*_^1^(*ε*_*f*_^*n*−1^(*g*))∨*f*, ∨ represents the pointwise maximum.

Morphological dilation and erosion operations apply a structuring element *B* including center element to an input image, constructing an output image with the same size. The shape and size of structuring element *B* determine the degree of dilation and erosion. The structuring element of size 3 × 3 is always exploited in dilation and erosion operation. If the size of *B* is 1 × 1, the output image is identical to the input image or else the output image will be dilated or eroded to a different degree according to the size of *B*.

The choice of mask images and marker images determines the reconstruction effect of an image. In general, if the raw noise image is selected as the mask image, the marker image is obtained by transforming the original noise image. In practical application, the marker image is always obtained by *g*=*ε*(*f*) or *g*=*δ*(*f*). This is because *ε*(*f*) ≤ *f* and *δ*(*f*) ≥ *f*, and they meet the condition of dilation and erosion operation.

Morphological opening and closing reconstructions are derived from the composition of morphological dilation and erosion reconstructions, which have a stronger filter capability.

Morphological opening operation firstly carries out morphological erosion operation on the image and then carries out morphological expansion operation on the image obtained by erosion operation. Morphological opening reconstruction, denoted by *R*^*O*^, is given as

(17) $$\begin{array}{c} R^{O}\left(f\right)=R_{R_{f}^{\varepsilon }\left(\delta \left(f\right)\right)}^{\delta }\left(\varepsilon \left(R_{f}^{\varepsilon }\left(\delta \left(f\right)\right)\right)\right). \end{array}$$

Morphological closing operation firstly carries out morphological expansion operation on the image and then carries out morphological erosion operation on the image obtained by expansion operation. Morphological closing reconstruction, denoted by *R*^*C*^, is depicted as

(18) $$\begin{array}{c} R^{C}\left(f\right)=R_{R_{f}^{\delta }\left(\varepsilon \left(f\right)\right)}^{\varepsilon }\left(\delta \left(R_{f}^{\delta }\left(\varepsilon \left(f\right)\right)\right)\right). \end{array}$$

Morphological opening reconstruction is suitable for accurately recovering the shape of the object after erosion, while the morphological closing reconstruction is more effective for smoothing the texture details. In this paper, we employ *R*^*C*^ to obtain reconstructed image due to the superiority of morphological closing reconstruction for texture detail smoothing.

## 3. Morphological Reconstruction-Based Improved FCM Clustering Algorithm with Guided Filter

In this section, we first propose a guided filter-based FCM with an influence factor, in which the influence factor *ρ* is set to adapt guidance image. Then we give the proof that the adjustment on guidance image is equal to changing parameter *ε*. Last, we propose the morphological reconstruction-based improved FCM clustering algorithm with guided filter.

### 3.1. A Guided Filter-Based FCM Method with an Influence Factor

Because the factor *ε* regarding guided filter in FCM + GF is defined as the scalar, the capability of FCM + GF to images in the case of various rate noise is weakening. To handle this issue, a guided filter-based fuzzy c-means method with an influence factor is proposed, in which a novel impact factor *ρ* is set to adapt the guidance image. The pseudocode of the IFCM_GF algorithm is depicted in Algorithm 1.

**Proof**

The parameter *ε* controls the ability of the guided filter to recognize “flat patch” and “high variance”, so *ε* should change with different noises in the image. Thus, we give the proof that multiplying the guidance image by an influence factor *ρ* is the same as changing parameter *ε* to *ε*/*ρ*^2^.

From (12) and (13), we can know that *a*_*k*_ and *b*_*k*_ associated with *ω*_*k*_ can be regarded as functions of parameter *ε*. Then, (12) and (13) can be rewritten as follows:

(19) $$\begin{array}{c} a{\left(\varepsilon \right)}_{k}=\frac{\left(1/\left|\omega \right|\right)\sum_{i\in \omega_{k}}I_{i}p_{i}-\mu_{k}\bar{p_{k}}}{\sigma_{k}^{2}+\varepsilon }, \end{array}$$

(20) $$\begin{array}{c} b{\left(\varepsilon \right)}_{k}=\bar{p_{k}}-a{\left(\varepsilon \right)}_{k}\mu_{k}. \end{array}$$

Then, the output *q*_*i*_ is defined as follows:

(21) $$\begin{array}{c} q{\left(\varepsilon \right)}_{i}=\frac{1}{\left|\omega \right|}\sum_{k:i\in \omega_{k}}\left(a{\left(\varepsilon \right)}_{k}I_{i}+b{\left(\varepsilon \right)}_{k}\right). \end{array}$$

Let the image *I*^*∗*^*ρ* be defined as the guidance image, the new linear coefficients *a*_*k*_′ and *b*_*k*_′ are computed as (22) and (23), respectively, and the new output *q*_*i*_′ is calculated as follows:

(22) $$\begin{array}{c} a_{k}^{\prime }=\frac{\left(1/\left|\omega \right|\right)\sum_{i\in \omega_{k}}I_{i}\rho p_{i}-\rho \mu_{k}\bar{p_{k}}}{\rho^{2}\sigma_{k}^{2}+\varepsilon }=\frac{1}{\rho }\frac{\left(1/\left|\omega \right|\right)\sum_{i\in \omega_{k}}I_{i}p_{i}-\mu_{k}\bar{p_{k}}}{\sigma_{k}^{2}+\left(\varepsilon /\rho^{2}\right)}. \end{array}$$

(23) $$\begin{array}{c} b_{k}^{\prime }=\bar{p_{k}}-a_{k}^{\prime }\rho \mu_{k}, \end{array}$$

(24) $$\begin{array}{c} q_{i}^{\prime }=\frac{1}{\left|\omega \right|}\sum_{k:i\in \omega_{k}}\left(a_{k}^{\prime }I_{i}\rho +b_{k}^{\prime }\right). \end{array}$$

Comparing (22) and (23) with (19) and (20), we can see that

(25) $$\begin{array}{c} a_{k}^{\prime }=\frac{1}{\rho }a{\left(\frac{\varepsilon }{\rho^{2}}\right)}_{k}, \end{array}$$

(26) $$\begin{array}{c} b_{k}^{\prime }=\bar{p_{k}}-a{\left(\frac{\varepsilon }{\rho^{2}}\right)}_{k}\mu_{k}=b{\left(\frac{\varepsilon }{\rho^{2}}\right)}_{k}. \end{array}$$

Embedding (25) and (26) into (24), we get

(27) $$\begin{array}{c} q_{i}^{\prime }=\frac{1}{\left|\omega \right|}\underset{k:i\in \omega_{k}}{\sum }\left(\frac{1}{\rho }a{\left(\frac{\varepsilon }{\rho^{2}}\right)}_{k}I_{i}\rho +b{\left(\frac{\varepsilon }{\rho^{2}}\right)}_{k}\right)=\frac{1}{\left|\omega \right|}\sum_{k:i\in \omega_{k}}\left(a{\left(\frac{\varepsilon }{\rho^{2}}\right)}_{k}I_{i}+b{\left(\frac{\varepsilon }{\rho^{2}}\right)}_{k}\right)=q{\left(\frac{\varepsilon }{\rho^{2}}\right)}_{i}. \end{array}$$

As shown in (27), the new output of the guided filter with guidance image *I∗ρ* is equal to the original output of the guided filter with parameter *ε*/*ρ*^2^. Therefore, adjusting the guidance image with an influence factor *ρ* is equivalent to changing parameter *ε*.

In this way, the proposed IFCM_GF method simplifies the selection of guiding filter parameters and improves the segmentation effect of different noise images.

### 3.2. Morphological Reconstruction-Based Improved FCM Clustering Algorithm with Guided Filter

The MRIFCM_GF clustering algorithm is developed in this subsection. Herein, by leveraging the morphological closing reconstruction, the reconstructed image *β* of the raw noise image *f* is firstly computed as follows:

(28) $$\begin{array}{c} \beta \;=\;R^{C}\left(f\right). \end{array}$$

Subsequently, FCM is employed to segment the reconstructed image and the guide filter is implemented on the membership matrix with the guidance of the raw noise image adjusted by *ρ*. The minimization problem of MRIFCM_GF is written as follows:

(29) $$\begin{array}{c} J_{MR}\left(U,V\right)=\sum_{c=1}^{C}\sum_{n=1}^{N}u_{cn}^{m}{\left\|\beta_{n}-\upsilon_{c}\right\|}^{2},\\ \begin{array}{cc} \text{subject to} & \sum_{c=1}^{C}u_{cn}=1,\;0<u_{cn}<1 \end{array}, \end{array}$$

where *β*_*n*_ denotes the *n-th* pixel of the reconstructed image *β*, *u*_*cn*_ indicates the membership of pixel *β*_*n*_ in cluster *c*, and *υ*_*c*_ means the prototype vector of cluster *c*.

The *U* matrix and *V* matrix are updated according to the following equations:

(30) $$\begin{array}{c} u_{cn}=\frac{1}{\sum_{j=1}^{C}{\left(\left\|\beta_{n}-\upsilon_{c}\right\|/\left\|\beta_{n}-\upsilon_{j}\right\|\right)}^{\left(2/\left(m-1\right)\right)a}}. \end{array}$$

(31) $$\begin{array}{c} \upsilon_{c}=\frac{\sum_{n=1}^{N}u_{cn}^{m}\beta_{n}}{\sum_{n=1}^{N}u_{cn}^{m}}, \end{array}$$

for 1 ≤ *c* ≤ *C*, 1 ≤ *n* ≤ *N*.

In each iteration, the guided filter is implemented on the membership metrics. The flowchart of the proposed MRIFCM_GF algorithm is shown in Figure 1. Firstly, input a noisy image to be segmented, reconstruct it by MR, and initialize cluster centers. Then, calculate memberships, adjust the guidance image by multiplying the influence factor, filter membership matrix by GF method, and update cluster centers iteratively until the stopping condition is satisfied. The pseudocode of the MRIFCM_GF algorithm is summarized in Algorithm 2.

By introducing the MR method, MRIFCM_GF solves the problem that IFCM_GF is not robust to different types of noisy images and high-noise images, and it is difficult to select influence factors when the noise ratio is unknown.

## 4. Experiments

The experiments are executed on synthetic images and Brain images. FCM [9], FCM + GF [17], FCM_S1 [12], FCM_S2 [12], and FRFCM [20] are selected for comparison analysis. The number of clusters is predetermined according to the prior information of the image to be clustered. The fuzzification index *m* is fixed to 2 and the error threshold *ξ* is defined as 10^−8^ in all methods. For FCM + GF, IFCM_GF, and MRIFCM_GF, the factor *ε* regarding guided filter is fixed to 0.1^4^, and the filtering window size is 3 × 3. For FCM_S1 and FCM_S2, *α* that trades off the influence of the neighbor term is set to 3.8, and the window size is 3 × 3. For IFCM_GF and MRIFCM_GF, the impact factors *ρ* are changed by various noise levels and types. For FRFCM and MRIFCM_GF, the mask image is the raw noise image, and a structuring element of size 3 × 3 is utilized to get the marker image.

### 4.1. Performance Measurement

The segmentation accuracy (SA) is adopted for quantitative comparison, and it is depicted as follows:

(32) $$\begin{array}{c} \text{SA}=\frac{D}{N}, \end{array}$$

where *D* means the number of properly clustered pixels and *N* indicates the whole number of pixels. All tested approaches are repeatedly conducted 100 times, so the average SA (ASA) is applied for comparative analysis.

### 4.2. Results on Synthetic Images

Two synthetic images, named ST and SF, respectively, are constructed artificially. The size of the ST image and SF image is 256 × 256. The ST image includes three classes, of which the intensities are 0, 85, and 170, respectively. The SF image is divided into four clusters, of which the intensities are 0, 85, 170, and 255, respectively. To examine the effectiveness of the presented algorithms for different noises, those synthetic images are corrupted by Gaussian noise and Salt & Pepper noise at various rates. The levels of Gaussian noise include 3%, 5%, 10%, and 15%. And the rates of Salt & Pepper noise contain 10%, 20%, and 30%.

Figure 2 illustrates the filtering results of MR, mean filter, and median filter on ST image with Gaussian noise (zero means and 5% variance) and Salt & Pepper noise (20% noise intensity). As shown in Figures 2(d) and 2(h), the median filter achieves a good denoising result on Salt & Pepper noise ST image, while it fails to remove Gaussian noise. At the same time, from Figures 2(c) and 2(g), it can be seen that the performance of the mean filter on the Gaussian noise ST image is slightly better than that of the median filter, but the mean filter performs worse on Salt & Pepper noise. The above observations denote that the mean filter and the median filter are sensitive to noise type. Conversely, as shown in Figures 2(b) and 2(f), the MR obtains excellent denoising results on both Gaussian noise image and Salt & Pepper image. This proves the ability of the MR to remove different type of noise.

Figure 3 shows the filtering results of MR and mean filter on ST image with various rate Gaussian noise. From Figures 3(i)–3(l), we can see that the denoising effects of the mean filter decrease with the increase of noise rate. In contrast, as shown in Figures 3(e)–3(h), the MR achieves good denoising results on all noise rates. The efficiency of the MR in denoising is helpful to get better segmentation results. More importantly, as the images with different noise rates are all well denoised by MR, they have similar grey level distributions, which are beneficial to simplify the selection of the influence factor in the MRIFCM_GF.

Figure 4 exhibits the segmentation results on the ST image with Gaussian noise (zero means and 5% variance).  Table 1 reflects the ASA of all testing methods on ST image with various noises. From Table 1, we can see that FCM obtains poor segmentation results on ST image due to its sensitivity to noise. Compared with the FCM, the FCM + GF achieves higher ASA. This reflects the superiority of the guided filter. But the improvement on ASA is very slight, which is because the fixed factor *ε* of the guided filter decreases the efficiency of FCM + GF. In contrast, by using an influence factor to adapt guidance image, the IFCM_GF can effectively segment different noise rate images and improve the segmentation results to some extent. This proves the benefit of the introduction of the influence factor *ρ*. When MRIFCM_GF is compared with IFCM_GF, we can see that the MRIFCM_GF achieves better ASA on image with Gaussian and high rate Salt & Pepper noise. This is because the MR can efficiently remove noise. Except the MRIFCM_GF, the other three methods (FCM_S1, FCM_S2, and FRFCM), which own the denoising operation, also get good ASA. However, FCM_S1 and FCM_S2 are greatly affected by the type of noise by virtue of the limitation of mean filter and median filter, and the FRFCM gets bad segmentation on edges. Different from FCM_S1, FCM_S2, and FRFCM algorithm, MRIFCM_GF obtains the best ASA on almost all ST images. This is because the introduced MR is effective in removing any type of noise, and the guided filter whose guidance image is adjusted by the influence factor can improve the segmentation on edges. From the segmented result of MRIFCM_GF (Figure 4(j)), we can see that the Gaussian noise is removed and the edge of the object is completely preserved.

Figure 5 reveals the ASA of the IFCM_GF with varying impact factors on ST images with various rate Gaussian noise. It can be seen that each curve makes a peak value; that is, no matter what the noise rate is, there is an optimal impact factor *ρ* which leads to the highest accuracy. What is more, the optimal impact factors at various noise rates change with a certain rule. It gets smaller with the increase in the noise rate. This finding is beneficial in the selection of *ρ* for the IFCM_GF if the noise rate of the image is known. However, it is challenging to know the noise rate of an image in advance, and the good influence factor values of different curves locate in different intervals, so it is not easy to select an appropriate *ρ* for IFCM_GF in practice.

Figure 6 shows the ASA of the MRIFCM_GF with different influence factors on ST images with various rate Gaussian noise. Firstly, we can see that the best value of *ρ* (0.014, 0.009, 0.008, and 0.005) still varies regularly. In addition, the curves of the 3% and 5% noise rate vary gently, which means the good value of *ρ* locates in a large scale. For example, as long as the value of *ρ* is set in interval (0, 0.1), the MRIFCM_GF will achieve high ASA on ST image with 3% rate Gaussian noise. What is more, when dealing with the image corrupted by high rate Gaussian noise, the good value of *ρ* is around zero. For instance, the good value of *ρ* of the MRIFCM_GF on 15% rate Gaussian noise image locates in interval (0, 0.008]. Therefore, a small *ρ* is appropriate for the MRIFCM_GF to segment an image with any rate Gaussian noise.

Table 2 presents the ASA of different methods on SF image with different rate Gaussian noises. We can see that the results obtained by different algorithms on SF images are similar to the ones on ST images. The performance of FCM deteriorates sharply as the noise rates increase. The FCM + GF and the IFCM_GF get higher ASA than FCM due to the employment of the guided filter. Moreover, the segmentation results of IFCM_GF are better than the ones of FCM + GF; this is because the IFCM_GF defines an impact factor *ρ* to adapt the guidance image. The MRIFCM_GF achieves the best ASA on all Gaussian noise images and high rate Salt & Pepper noise images. This is another proof of the superiority of the combination of the MR and the guided filter.

Figure 7 displays the segmentation results of tested models on SF image with Gaussian noise (zero means and 5% variance). As shown in Figures 7(d)–7(h), the FCM, the FCM_S1, the FCM_S2, the FCM + GF, and the IFCM_GF suffer from the noise, which leads to numerous misclassifications. From Figures 7(i) and 7(j), it can be seen that there are a few noise points remaining in the segmentation results of the FRFCM and MRIFCM_GF. What is more, the MRIFCM_GF obtains better performances on the edges than the FRFCM.

Figures 8 and 9 show the ASA of the IFCM_GF and the MRIFCM_GF with various impact factors on SF images corrupted by Gaussian noise. From Figure 8, it can be seen that the best impact factor of the IFCM_GF on different rate Gaussian noise does not vary regularly. What is more, the values of the good influence factors on different noise rates locate in various intervals. For example, the good influence factor interval of the 5% noise rate is [0.03, 0.049]; meanwhile, the one of the 15% noise rate is [0.008, 0.027]. Thus, it is difficult to choose an appropriate influence factor for the IFCM_GF without knowing the noise rate. On the contrary, as shown in Figure 9, the best influence factors of the MRIFCM_GF on the SF images with Gaussian noise decrease regularly as the noise rates change. In addition, the good influence factor of the MRIFCM_GF on a noise rate is also adapted to another noise rate. For instance, if the influence factor is set to 0.005, the ASA of MRIFCM_GF on SF image with 3% Gaussian noise is 0.9984, and the one on 15% Gaussian noise image is 0.9845. In summary, it is easy to set the influence factor *ρ* for the MRIFCM_GF.

## 5. Results on Brain Images

To further verify the advantage of the MRIFCM_GF, the brain magnetic resonance images (Brian images) collected from “BrainWeb” [21] are considered as the test images in this subsection. The size of the Brain images is 181 × 217. Brain images are corrupted by Rician noise, and the noise rates include 5%, 10%, 15%, 20%, and 25%.

The segmentation results of tested algorithms on Brain image with 5% Rician noise are illustrated in Figure 10.  Table 3 details the ASA of all methods on the Brain image with Rician noise. When the noise rate is 5%, the IFCM_GF, the FCM + GF, and the FCM achieve the best three results (0.9999, 0.9998, and 0.9993 on ASA, resp.). This is because the 5% Rician noise has little influence on image segmentation, and the denoising operations (mean filter, median filter, and the MR) are not helpful in this case but only lead to the destruction of the image edges. However, with the increase of noise rate, the methods with denoising operations get better ASA. For example, when the noise rate is 10%, the FCM_S1, the MRIFCM_GF, and the FCM_S2 get the best three results on ASA (0.9866, 0.9844, and 0.9722, resp.). More importantly, the proposed MRIFCM_GF method obtains the best ASA when the noise rate is high (15%, 20%, and 25%). The excellent performance of the MRIFCM_GF results from both the ability of the MR to remove heavy noise and the superiority of the influence factor to enhance the capacity of the guided filter to reserve edges.

Figures 11 and 12 present the ASA of IFCM_GF and MRIFCM_GF with different influence factors on Brain images. As shown in Figure 11, for the IFCM_GF, the good values of the influence factor *ρ* for different noise rates locate in different intervals. For instance, the good influence factor values for 10% Rician noise Brain image locate in [0.13, 0.2]; meanwhile, the ones for 25% Rician noise Brain image locate in [0.01, 0.04]. So, it is challenging to set the value of the influence factor *ρ* for the IFCM_GF without knowing the noise rate. On the contrary, from Figure 12, we can see that the good influence factor values of the MRIFCM_GF on images with different rate noises locate in the same interval. Specifically, if only the value of *ρ* is set larger than 0.06, the MRIFCM_GF can obtain good ASA on all Brain images whatever the noise rate is.

## 6. Conclusions

In this paper, we first present the IFCM_GF method, in which a novel impact factor *ρ* is designed to adapt the guidance image. The essence of this adjustment on guidance image is proved to be equal to the change on parameter *ε* of guided filter. IFCM_GF improves the segmentation performance of images with various noise rates by varying the value of *ρ*. Thus, to reinforce the heavy noise image segmentation quality and simplify the selection of impact factor, we further propose the MRIFCM_GF algorithm, in which the original noise image is reconstructed by MR before clustering. The MR is effective in removing noise ignoring noise type, so the MRIFCM_GF achieves better performance than the IFCM_GF. More importantly, the MR can efficiently remove any rate noise and the reconstructed images of different rate noise images have similar grey distributions, so it is easy to set an appropriate influence factor for the MRIFCM_GF without knowing noise rates.

In the future, we will explore how to automatically get an appropriate influence factor *ρ* based on the type and rate of noise. Moreover, the choice of mask image and marker image determines the reconstruction result, so we will continue to study how to select mask or marker image in MR to obtain better performance.

## Figures and Tables

**Figure 1:** The block diagram of the overall methodology of the MRIFCM_GF algorithm.

**Figure 2:** The filter results of tested models on different noise images. (a) Gaussian noise image (zero means and 5% variance). (b) Filtering result of MR on (a). (c) Filtering result of mean filter on (a). (d) Filtering result of median filter on (a). (e) Salt & Pepper noise image (20% noise intensity). (f) Filtering result of MR on (e). (g) Filtering result of mean filter on (e). (h) Filtering result of median filter on (e).

**Figure 3:** The filtering results of MR and mean filter on ST image with various rates of Gaussian noise. (a) Gaussian noise image (zero means and 3% variance). (b) Gaussian noise image (zero means and 5% variance). (c) Gaussian noise image (zero means and 10% variance). (d) Gaussian noise image (zero means and 15% variance). (e) Filtering result of MR on (a). (f) Filtering result of MR on (b). (g) Filtering result of MR on (c). (h) Filtering result of MR on (d). (i) Filtering result of mean filter on (a). (j) Filtering result of mean filter on (b). (k) Filtering result of mean filter on (c). (l) Filtering result of mean filter on (d).

**Figure 4:** The segmentation results on ST image with Gaussian noise (zero mean and 5% variance). (a) Ground truth. (b) Raw noise image. (c) Reconstructed image of raw noise image. (d) FCM. (e) FCM_S1. (f) FCM_S2. (g) FCM + GF. (h) IFCM_GF. (i) FRFCM. (j) MRIFCM_GF.

**Figure 5:** The ASA of IFCM_GF with various impact factors on ST images corrupted by varying levels of Gaussian noise.

**Figure 6:** The ASA of MRIFCM_GF with various impact factors on ST images corrupted by varying levels of Gaussian noise.

**Figure 7:** The segmentation results on SF image with Gaussian noise. (a) Ground truth. (b) Raw noise image (zero mean and 5% variance). (c) Reconstructed image of raw noise image. (d) FCM. (e) FCM_S1. (f) FCM_S2. (g) FCM + GF. (h) IFCM_GF. (i) FRFCM. (j) MRIFCM_GF.

**Figure 8:** The ASA of IFCM_GF with various impact factors on SF images corrupted by varying levels of Gaussian noise.

**Figure 9:** The ASA of MRIFCM_GF with various impact factors on SF images corrupted by varying levels of Gaussian noise.

**Figure 10:** The segmentation results on Brain image. (a) Ground truth. (b) Raw noise image (Rician noise intensity is 15%). (c) Reconstructed image of raw noise image. (d) FCM. (e) FCM_S1. (f) FCM_S2. (g) FCM + GF. (h) IFCM_GF. (i) FRFCM. (j) MRIFCM_GF.

**Figure 11:** The ASA of IFCM_GF with various influence factors corrupted by varying levels of Rician noise rate.

**Figure 12:** The ASA of MRIFCM_GF with various influence factors corrupted by varying levels of Rician noise rate.

**Algorithm 1:** IFCM_GF algorithm.

**Algorithm 2:** MRIFCM_GF algorithm.

**Table 1:** The ASA of tested algorithms on ST images with various noises.

Noise		FCM	FCM_S1	FCM_S2	FCM + GF (*ε*=0.1^4^)	IFCM_GF (*ρ*)	FRFCM	MRIFCM_GF (*ρ*)
3% Gaussian	0.7028		0.9783	0.9742	0.6984	0.7520 (0.047)	0.9982	^*∗*^ **0.9993 (0.014)**
5% Gaussian	0.6471		0.9166	0.8716	0.6646	0.7166 (0.034)	0.9965	^*∗*^ **0.9987 (0.009)**
10% Gaussian	0.5806		0.7628	0.7497	0.6172	0.7153 (0.02)	0.9892	^*∗*^ **0.9964 (0.008)**
15% Gaussian	0.5499		0.7292	0.7139	0.5924	0.7082 (0.017)	0.9425	^*∗*^ **0.9907 (0.005)**
10% Salt & Pepper	0.9431		0.9389	0.9826	0.9443	^*∗*^ **0.9995 (0.008)**	0.9991	0.9993 (0.009)
20% Salt & Pepper	0.8873		0.8757	0.9647	0.8916	^*∗*^ **0.9993 (0.006)**	0.9989	^*∗*^ **0.9993 (0.004)**
30% Salt & Pepper	0.8304		0.7806	0.9409	0.8366	0.9981 (0.002)	0.9976	^*∗*^ **0.9982 (0.003)**

^*∗*^The best segmentation accuracy among the group.

**Table 2:** The ASA of tested algorithms on SF images with various noises.

Noise	FCM	FCM_S1	FCM_S2	FCM + GF (*ε*=0.1^4^)	IFCM_GF (*ρ*)	FRFCM	MRIFCM_GF (*ρ*)
3% Gaussian	0.7277	0.9716	0.9736	0.7333	0.9274 (0.02)	0.9972	^*∗*^ **0.9986 (0.019)**
5% Gaussian	0.6417	0.9301	0.9271	0.6486	0.7492 (0.04)	0.9952	^*∗*^ **0.9979 (0.016)**
10% Gaussian	0.5392	0.8103	0.8003	0.5250	0.6132 (0.002)	0.9857	^*∗*^ **0.9944 (0.004)**
15% Gaussian	0.4902	0.7331	0.7348	0.4709	0.5620 (0.015)	0.9592	^*∗*^ **0.9847 (0.001)**
10% Salt & Pepper	0.9233	0.9329	0.9746	0.9273	^*∗*^ **0.9995 (0.003)**	0.9990	0.9994 (0.007)
20% Salt & Pepper	0.8475	0.8617	0.9477	0.8620	^*∗*^ **0.9989 (0.002)**	0.9982	^*∗*^ **0.9989 (0.005)**
30% Salt & Pepper	0.7708	0.7613	0.9152	0.7958	0.9973 (0.001)	0.9966	^*∗*^ **0.9975 (0.003)**

^*∗*^The best segmentation accuracy among the group.

**Table 3:** The ASA of tested algorithms with various noises on Brain images.

Noise	FCM	FCM_S1	FCM_S2	FCM + G (*ε* = 0.1^4^)	IFCM_GF (*ρ*)	FRFCM	MRIFCM_GF (*ρ*)
5% Rician	0.9993	0.9953	0.9908	0.9998	^*∗*^ **0.9999 (0.15)**	0.9837	0.9952 (0.14)
10% Rician	0.8427	^*∗*^ **0.9866**	0.9772	0.8480	0.9380 (0.15)	0.9762	0.9844 (0.1)
15% Rician	0.7075	0.9085	0.8313	0.7265	0.8167 (0.05)	0.9387	^*∗*^ **0.9483 (0.08)**
20% Rician	0.6240	0.7993	0.7823	0.6456	0.7731 (0.03)	0.8984	^*∗*^ **0.9152 (0.08)**
25% Rician	0.5540	0.7674	0.7477	0.5862	0.7410 (0.02)	0.8631	^*∗*^ **0.8745 (0.07)**

^*∗*^The best segmentation accuracy among the group.

## Data Availability

Data used to support the study were obtained from public datasets (BrainWeb, https://brainweb.bic.mni.mcgill.ca/brainweb/).
